RETRACTED

# Synthesis, Optical and Structural Properties of Copper Sulfide Nanocrystals from Single Molecule Precursors

**DOI:** 10.3390/nano7020032

**Published:** 2017-02-04

**Authors:** Peter A. Ajibade, Nandipha L. Botha

**Affiliations:** Department of Chemistry, University of Fort Hare, Private Bag X1314, Alice 5700, South Africa; 200904696@ufh.ac.za

**Keywords:** CuS, dithiocarbamate, nanoparticles, electron microscopy, atomic force microscopy (AFM)

## Abstract

We report the synthesis and structural studies of copper sulfide nanocrystals from copper (II) dithiocarbamate single molecule precursors. The precursors were thermolysed in hexadecylamine (HDA) to prepare HDA-capped CuS nanocrystals. The optical properties of the nanocrystals studied using UV–visible and photoluminescence spectroscopy showed absorption band edges at 287 nm that are blue shifted, and the photoluminescence spectra show emission curves that are red-shifted with respect to the absorption band edges. These shifts are as a result of the small crystallite sizes of the nanoparticles leading to quantum size effects. The structural studies were carried out using powder X-ray diffraction (XRD), transmission electron microscopy (TEM), scanning electron microscopy (SEM), energy dispersive X-ray spectroscopy (EDS), and atomic force microscopy. The XRD patterns indicates that the CuS nanocrystals are in hexagonal covellite crystalline phases with estimated particles sizes of 17.3–18.6 nm. The TEM images showed particles with almost spherical or rod shapes, with average crystallite sizes of 3–9.8 nm. SEM images showed morphology with ball-like microspheres on the surfaces, and EDS spectra confirmed the presence of CuS nanoparticles.

## 1. Introduction

The synthesis and studies of the optical and structural properties of nanomaterials expecially metal chalcogenides have received considerable attention in the last decades due to quantum confirement effects associated with their small crystallites sizes [1,2,3,4,5,6] that give them novel properties that make them useful in light-emitting diodes [7], solar cells [8], fuel cells [9], drug delivery [10,11], and as catalysts for industrial transformations [12,13,14,15,16]. Group 12 chalcogenides—especially ZnS [17,18] and CdS [19,20] nanoparticles have been widely studied but their toxicity limits any possible applications. As of result of the inherent toxicity of group 12 metal chalcogenides, copper sulfide nanocrystals are being explored for different applications [21,22,23,24,25,26,27]. CuS nanoparticle are also attractive because they exist in different stoichiometric compositions with varying crystalline phases [28,29,30,31].

Several methods have been used to synthesize metal sulfide nanoparticles, including solvothermal synthesis [32], microwave [33], ultrasonic irradiation [34], and thermolysis of single-source precursors in high boiling point solvents that act as surface passivating agents [35,36,37,38]. For the synthesis of CuS nanocrystals, different synthetic techniques have also been used [39,40,41,42] to produce nanoparticles with varying morphologies such as nanotubes [43], nanowires [44], and nanoplatelets [45], among others [46,47]. Among nanocrystal synthetic methods, the single-source precursor technique produces nanocrystals with reasonable monodispersity [48], and studies have indicated that the sizes and shapes of the resulting nanocrystals are influenced by the precursor concentration [49], reaction time [50], and temperature [51]. As a result of nanocrystals’ unique size-dependent physical and chemical properties [52,53], the synthesis of monodisperse nanocrystals continue to attract much research attention [54]. In this paper, we report the use of three copper (II) dithiocarbamate complexes as efficient single-source precursors for the preparation of hexadecylamine (HDA)-capped copper sulfides nanoparticles. HDA was used as capping agent to passivate the sulface of the nanoparticles and prevent the particles from forming clump to larger particles. The optical and structural properties of the nanoparticles were studied using UV–visible, photoluminescence (PL), X-ray diffraction (XRD), transmission electron microscopy (TEM), scanning electron microscopy (SEM), energy dispersive X-ray spectroscopy (EDS) and atomic force microscopy (AFM).

RETRACTED

## 2. Materials Methods

### 2.1. Materials and Physical Measurements

All chemicals and reagents were used as received without further purifications. Hexadecylamine (HDA), trioctylphosphine (TOP), toluene, and methanol are analytical-grade reagents used as obtained from Sigma-Aldrich (St. Louis, MO, USA). The ligands, sodium salt of *N*-phenyldithiocarbamate, *N*-ethylphenyldithiocarbamate, and morpholinedithiocarbamate were prepared using literature procedures [55,56]. Powder X-ray diffraction patterns were obtained from Bruker D8 Advance (Billerica, MA, USA) equipped with a proportional counter using Cu Kα radiation (λ = 1.5405 Å, nickel filter). TEM images were obtained from a ZEISS Libra 120 electron microscope (Oberkochen, Germany). Thermogravimetric analysis (TGA) was recorded on an SDTQ 600 thermogravimetric instrument (New Castle, DE, USA). The infrared spectra were obtained from a PerkinElmer Paragon 2000 Fourier-transform infrared (FTIR) spectrophotometer (Waltham, MA, USA) using the KBr disk method, UV–vis spectra were recorded on a PerkinElmer Lambda 25 UV–vis spectrophotometer (Waltham, MA, USA), and the photoluminescence study was recorded with PerkinElmer LS 45 fluorimeter (Waltham, MA, USA) (SEM was done using Jeol JSM-6390 LVSEM (Akishimo, Tokyo, Japan) at a rating voltage of 15–20 kV at different magnifications, as indicated on the SEM images. Energy dispersive spectra were processed using EDS attached to a Jeol, JSM-6390 LV SEM with Noran System *Six* software (Waltham, MA, USA). AFM was carried out using Digital Instruments Nanoscope, Veeco, MMAFMLN-AM (Multimode) (San Jose, CA, USA).

RETRACTED

### 2.2. Synthesis of Copper (II) Dithiocarbamate Complexes

In a typical synthesis, a solution of CuCl_2_ (0.625 mmol) was dissolved in 25 mL of water or methanol and added to 1.250 mmol of the sodium salt of *N*-phenyldithiocarbamate. Greenish brown precipitates formed immediately and the reaction mixture was stirred for 1 h at room temperature. The products were filtered and washed several times with water and methanol. The resulting copper (II)-*N*-phenyl dithiocarbamate complex [Cu(phendtc)_2_] was dried at room temperature. A similar procedure was used for the synthesis of copper (II) complexes of *N,N’*-ethylphenyldithiocarbamate [Cu(ephendtc)_2_] and morpholinedithiocarbamate [Cu(morpdtc)_2_].

[**Cu(phendtc)_2_**]: Selected IR (cm^−1^): *v*(N–H) 3451, *v*(C–N) 1450, *v*(C–S) 1109, *v*(M–S) 328.

[**Cu(ephendtc)_2_**]**:** Selected IR (cm^−1^): *v*(N–H) 3417, *v*(C–N) 1472, *v*(C–S) 1067, *v*(M–S) 329.

[**Cu(morpdtc)_2_**]**:** Selected IR (cm^−1^): *v*(N–H) 3416, *v*(C–N) 1484, *v*(C–S) 1016, *v*(M–S) 327.

### 2.3. Synthesis of HDA-Capped CuS Nanoparticles

The metal sulfide nanoparticles were prepared by dissolving 0.20 g of each metal complex in 4 mL of TOP and injected into 3 g of hot HDA at 180 °C. An initial decrease of about 20–30 °C in temperature was observed. The solution was stabilized at 180 °C and the reaction continued for 1 h. After completion, the reaction mixture was allowed to cool to 70 °C, and methanol was added to precipitate the nanoparticles. The solid was separated by centrifugation and washed three times with methanol. The resulting solid precipitates of HDA-capped copper sulfide nanoparticles were dispersed in toluene for further analysis. Synthesized CuS nanoparticles from copper (II) *N*-phenyldithiocarbamate complex is labeled **CuS1**; from copper (II) *N*,*N*-ethyl phenyldithiocarbamate complex is labeled **CuS2**, and from copper (II) morpholinedithiocarbamate complex is labeled **CuS3**.

## 3. Results and Discussion

### 3.1. Optical Properties of the CuS Nanoparticles

UV–vis spectrophotometry was used to study the absorption properties of the as-prepared nanoparticles. Figure 1 shows the absorption spectra of the CuS nanoparticles and reveals that the absorption band edges of **CuS1** and **CuS2** are almost similar and appear at about 287 nm. The absorption spectrum of **CuS3** differs slightly from the other two, with an absorption band edge at about 286 nm. The absorption spectra showed considerable blue-shift, which could be ascribed to the quantum size effect of the nanoparticles due to their smaller crystallite sizes [57,58]. The optical properties of semiconductor nanoparticles are strongly influenced by their crystallite sizes and shapes [59,60,61,62]. The calculated band gap energies for **CuS1** and **CuS2** are 4.33 eV. This value is greater than that of the bulk CuS, which is 1.2 eV [39]. **CuS3**, with absorption maxima at 286 nm and calculated band gap energy of 4.3 eV, is also blue-shifted and quantum confined. Figure 2 shows the photoluminescence spectra of the as-prepared CuS nanoparticles obtained at room temperature. The spectra are red-shifted intense but narrow-peaked at 620 nm. The observed red-shift could be attributed to the trap-related electron-hole recombination [51,52]. The spectra show that nanoparticles obtained from different precursors have the same emission maxima but differ in their intensity and peak widths. **CuS2** prepared from (Cu(ephendtc)_2_) shows a narrow and sharp emission peak that is higher than the other two, indicating better electronic passivation of the **CuS2** nanoparticles by the capping agents. The reduced broadness of the emission curves can be attributed to their narrow size distributions. Although the absorption spectrum of **CuS3** is different from those of **CuS1** and **CuS2**, the emission spectra of the three nanoparticles are similar, differing only in their intensities.

RETRACTED

### 3.2. Powder X-Ray Diffraction Analysis of the CuS Nanoparticles

XRD patterns for the nanocrystals prepared using different precursors are shown in Figure 3. The diffraction patterns showed four broad peaks that could be indexed to the hexagonal covellite crystalline phase of CuS with characteristic (101), (102), (103), and (006), and in good agreement with the standard data for CuS (JCPDS Card No. 06-0464) [63,64]. The average crystallite size of the nanoparticles, as estimated using Scherrer equation [65], are 18.09 nm for **CuS1**, 17.3 nm for **CuS2**, and 18.6 nm for **CuS3**, respectively.

### 3.3. Morphology of the CuS Nanocrystals

The morphology and microstructure of the as-prepared CuS nanocrystals were studied with TEM, SEM, EDS, and AFM analyses. Figure 4 shows TEM images of the HDA-capped copper sulfide nanoparticles, which vary in shape from rodlike in **CuS1** to almost spherical and fairly monodispersed in **CuS2** and **CuS3**. The TEM image of **CuS1** shows copper sulfide nanoparticles with the average crystal size in the range of 5.10–9.80 nm, and its shapes appears to be a mixture of rodlike and some cubic-shaped nanoparticles. The TEM image of **CuS2** shows nanoparticles that are small, spherically shaped particles which are uniformly distributed, with the average crystallite size in the range 3.06–4.35 nm. The TEM image of **CuS3** shows small, spherically shaped nanoparticles with some aggregation. The crystallite sizes of the nanoparticles are in the range 3.02–4.32 nm.

The SEM images of the CuS nanoparticles and their elemental composition, as confirmed by EDS, are shown in Figure 5. It can be seen that the surface of the particles appears smooth with small microspheres on the surface. As expected, the microspheres on the surface are much bigger than that of the crystallite size measured by TEM analysis. This may be due to the agglomeration of crystallites occurring in the course of preparing the sample for SEM analyses. The EDS patterns show copper and sulfur, confirming the formation of CuS nanoparticles. Other peaks that seems to be common for all XRD spectra are phosphorus, nitrogen, and oxygen due to TOP that was used for dispersing the precursor and the HDA that was used as a capping agent.

AFM was used to investigate the surface morphology and surface roughness [66,67]. AFM techniques provide microscopic and topographic information about the surface relief of the nanocrystals [67,68]. Thus, digital images for quantitative measurements of surface features such as three-dimensional simulation, average roughness (*R*a), and root mean square roughness (*R*q) can be obtained by AFM [66,67,68,69]. The topographical view of the nanoparticles (Figure 6, Figure 7 and Figure 8) reveals that **CuS1** and **CuS3** nanoparticles are richer in dents and irregular surfaces than **CuS2**. The values of *R*q and *R*a were found to be 5.77 and 2.76 nm for **CuS1**; 24.8 and 18.9 nm for **CuS2**; and 12.6 and 9.00 nm for **CuS3**, respectively.

## 4. Conclusions

Copper (II) complexes of dithiocarbamate were used as single-source precursors to synthesize HDA-capped CuS nanoparticles. The optical studies showed that the absorption spectra of the as-prepared nanoparticles are blue-shifted and the emission maxima showed a narrower size distribution, which indicates a size quantum effect. The XRD patterns were indexed to the hexagonal CuS nanocrystals with estimated particle sizes of 17.3–18.6 nm. TEM images showed nanoparticles that are almost spherical in shape and fairly monodispersed, with average crystallite sizes of 3–9.8 nm.

RETRACTED

## Figures and Tables

**Figure 1:** Absorption spectra of copper (II)-*N*-phenyl dithiocarbamate complex (**CuS1**), copper (II)-*N*,*N*-ethylphenyldithiocarbamate (**CuS2**), and copper (II)-morpholinedithiocarbamate (**CuS3**) nanoparticles.

**Figure 2:** Emission spectra of **CuS1**, **CuS2**, and **CuS3** nanoparticles.

**Figure 3:** Powder X-ray diffraction (XRD) patterns of **CuS1** (**A**), **CuS2** (**B**), and **CuS3** (**C**) nanoparticles * hexadecylamine (HDA).

**Figure 4:** Transmission electron microscopy (TEM) images of **CuS1** (**A**), **CuS2** (**B**), and **CuS3** (**C**) nanoparticles.

**Figure 5:** Scanning electron microscopy (SEM) images of **CuS1**, **CuS2**, and **CuS3** nanoparticles.

**Figure 6:** Atomic force microscopy (AFM) surface roughness (**A**) and 3D topographical images (**B**) of **CuS1** nanoparticles.

**Figure 7:** AFM surface roughness (**A**) and 3D topographical images (**B**) of **CuS2** nanoparticles.

**Figure 8:** AFM surface roughness (**A**) and 3D topographical images (**B**) of CuS3 nanoparticles.
